The article "Analysis of Internet Public Opinion Popularity Trend Based on a Deep Neural Network" was published in 2022. Journal: Comput Intell Neurosci.

# Analysis of Internet Public Opinion Popularity Trend Based on a Deep Neural Network

**DOI:** 10.1155/2022/9034773

**Published:** 2022-07-06

**Authors:** Min Gong

**Affiliations:** King's College London, London WC2R 2LS, UK

## Abstract

In the context dominated by Internet communication, people's various emotions can be clearly reflected through network public opinion, whether it is the view of political affairs, the preference for entertainment, or the demand for life. This also allows management or providers to meet their needs more specifically. Based on today's need to understand the trend of Internet public opinion, this paper describes a deep neural network (DNN). A deep neural network is a machine learning model that is the foundation of deep learning and has a strong ability to mine potential information in data. By improving the loss function of the neural network, this paper reduces the influence of unbalanced data on the classification results and improves the classification effect of the model on a small number of categories. Aiming at the different lengths of Internet text, a more robust model of text sentiment classification is proposed, which makes the HCB-Att model better extract the local information and contextual information of the text. Finally, through comparative experiments, the optimization model used in this paper is proved to be effective for the analysis of network public opinion sentiment.

## 1. Introduction

Deep belief network prediction training algorithms are a robust and useful method for generating deep neural networks, optimizing, and reducing generalization errors. We use this algorithm for speech recognition in a large vocabulary context, and the model has made recent advances in telephone recognition using deep belief networks. It describes the key components of the model by applying CD-DNN-HMM to the LVSR acquisition process and analyzes the impact of various modeling options on performance [1]. This paper provides an entry point for interpreting deep neural network models and for interpreting their predictions. It is based on the tutorial given on the ICASSP 2017. There is a huge need for improved Reynolds mean turbulence models, informed by a richer set of turbulence physics, that can represent a richer turbulence physics. In this paper, we propose a method to learn a Reynolds stress anisotropy tensor model from simulation data with high fidelity using deep neural networks. We propose a new neural network architecture that beds Galileo invariance into the predicted anisotropic tensor using a multiplication layer with an invariant tensor basis. This Reynolds stress anisotropy prediction of the invariant neural network is propagated to the velocity field of the two test cases [2]. During the DNN learning process, large training sets ensure powerful modeling capabilities to estimate complex nonlinear mappings from observed noisy speech to desired clean signals. The acoustic context was found to improve the continuity of speech, successfully separating it from background noise without the annoying musical artifacts common to traditional speech enhancement algorithms. A series of pilot experiments were conducted under multicondition training and simulating voice data for more than 100 hours. In addition, in an assessment of subjective preferences of 10 listeners, it was found that 76.35% of subjects preferred DNN-based enhanced speech over voice obtained using other traditional techniques [3]. In view of the frequent occurrence of network public opinion on the Internet, this paper analyzes the requirements and business processes of the network public opinion monitoring and analysis system. This paper introduces the five-tier architecture of the information monitoring and analysis system, including automatic information collection, information preprocessing, information database, information analysis and service, information visualization, and reporting. Then, the implementation of key technologies in the system is studied, including public opinion information collection technology, information search analysis, information search and cluster analysis, speech analysis, and trend prediction analysis [4]. Compared with the original system, the accuracy of topic extraction and public opinion trend prediction of the redesigned system has been significantly improved, which further verifies the correctness of the scheme. A new model is built to describe public opinion events that change in thermal trends. The results show that the model can simulate the hot trend of public opinion events. It provides a quantitative basis for the government to control and guide public opinion and development plans. Audio messages, video messages, and facial expression messages are inversely correlated with new media information preferences. The volume is indexed by repeated questions in polls as well as variations of these questions. These questions came from the U.S. national sample conducted by the AIPO (Gallup), NORC, and Roper (mainly the general population) and have been conducted in the Roper Archived by the Center for Public Opinion Research. More than 90% of the basic data for the survey is only available from the Roper Center. The index was first surveyed in September 1936, the most recent in October 1973. The purpose of the index is to build a database for measuring and analyzing social change. 70 main topics include specific research questions from trends in agricultural farm incomes to U.S. attitudes toward Yugoslavia. Each item includes the wording of the question, the investigative body that raised the question, the number and date of the investigation, and the number of questions [5]. Social media, as an adjunct to researchers, have become an important communication channel for public opinion because of their popularity and rapid communication ability because they serve as the main virtual space to raise new public issues, discuss these issues, and put forward opinions on these issues. With the recognition of the importance of social media, many businesses and governments have tried to use social media as a marketing tool or a public opinion perception tool. In the aftermath of the Fukushima disaster, nuclear power has become one of the hot public issues in South Korea. Nuclear power is a double-edged sword because it is currently the most efficient way to generate electricity, and there are potential risks, such as radiation leakage. Governments and policymakers need to constantly monitor public perceptions of nuclear power, as they may change depending on the events [6]. In this study, we aim to propose a method to sense the public perception of nuclear power and analyze its trends based on public opinion mining techniques. We have also proposed a measure to track changes in the direction of public opinion on nuclear power. To demonstrate the utility of the proposed method, we collected tweets from South Korea Nuclear Power in 2009 and 2013. After categorizing tweets in 2009 and 2011, an emotional dictionary containing both positive and negative terms was constructed. Performance tests conducted using tweets in 2012 and 2013 showed that the method could be applied in practice. [7]. The social network Weibo's opinion research on Chinese medicine during the epidemic in novel coronavirus pneumonia (novel coronavirus pneumonia) comprehensively considers the research background of the people's fight against novel coronavirus pneumonia and the power of Chinese medicine during the epidemic to determine the research theme and research object. The timeline is divided into three stages based on the overall thermal change. In order to explore and compare people's emotions and concerns about TCM in different stages, deep learning analysis methods such as sentiment analysis and latent Dirichlet distribution analysis are used for large flow of people. The study found that the public's positive “emotional component” towards TCM increased significantly on the timeline. At the same time, the public's autonomy has increased, and overall public opinion has begun to show an upward trend [8]. The whole society pays great attention to it. With the continuous development of Internet technology, especially the advent of the self-media era, public opinion, as a public force, has brought a comprehensive impact and new challenges to the management of the college entrance examination. When disseminating public opinion on the college entrance examination, the organs of the college entrance examination shall understand and study the role and discipline of the media. Learn to contact the media and cooperate for win-win results. Build good relationships with media resources and networks. Adhere to the problem-oriented, and actively build a professional public opinion response mechanism. In particular, the focus is on the disposal in the context of new media public opinion. Facts have proved that timely, reasonable, and appropriate response is the crux of public opinion response and crisis management [9]. It can predict the heat of public opinion, proactively guide public opinion in time, and let the public accept and form a positive cognitive impression, which is conducive to the healthy development of public opinion. In this paper, the staging factor is introduced into the wheel selection method of the artificial swarm algorithm to improve the global search ability of ABC and to predict the hot trend of network public opinion based on the improved ABC-BP model. This model has a higher prediction accuracy when compared to other models. The above theoretical research can provide an effective model for the government and enterprises to timely grasp the hot trend of online public opinion and provide a reference for formulating feasible guidance measures and marketing strategies and added up to obtain the predicted values of raw data. Finally, to account for the accuracy and validity of the EEMD-NAR model [10], a new model is built to describe public opinion events that change in thermal trends. The results show that the model can simulate the hot trend of public opinion events. In the past era, with the explosive interaction and dissemination of Internet information, collecting a large amount of Internet information and mining hot topics of network public opinion have become a hot branch of research. In this paper, a neural network (NN) based network public opinion evaluation model and prototype are proposed. First of all, a new evaluation index system is proposed and designed. Subsequently, we proposed a new poll analysis evaluation model and discussed the detailed steps. Finally, we conducted experiments to test the robustness and effectiveness of the method, and then we proposed a detailed explanation. As the number of Weibo users increases, the platform generates a large amount of data every day [11]. The rapid spread of data will lead to widespread changes in public opinion. Therefore, to correctly predict the public opinion on Weibo is an urgent challenge. To this end, this paper proposes a method to predict microblog public opinion using improved BP. First of all, according to the characteristics of the microblog public opinion, this paper constructs 9 public opinion indicators to analyze microblog public opinion. Third, since BP is susceptible to initial weight selection and shows a poor convergence rate, a genetic algorithm is introduced to optimize BP. However, genetic algorithms can easily fall into local optimal solutions [12]. Therefore, using the urban acceptance criterion to improve the local search capability of genetic algorithms, we propose an IGABP algorithm based on improved genetic algorithms. Finally, the effectiveness of the IGABP algorithm is verified by extracting and normalizing microblog data. Experimental results show that the IGABP algorithm is feasible in the prediction process [13]. The establishment of an effective network public opinion risk early warning index system and the evaluation method is an important basis for an emergency decision. Automated and rapid online poll assessments can greatly reduce human output. In order to establish an evaluation method suitable for the development level of network public opinion, a comprehensive evaluation algorithm combining the BP neural network and hierarchical analysis (AHP) is proposed. Besides, the possible optimization method is also discussed [14].

## 2. Key Technologies for Event Analysis

### 2.1. Event Recognition Technology

#### 2.1.1. Hierarchical Clustering

Hierarchical clustering is a clustering algorithm that divides datasets into different levels based on the distance between clusters, resulting in a tree-shaped clustering structure. Depending on the division strategy, it can be divided into “top-down” and “bottom-up” [15].

Common calculation formulas for measuring distances between clusters are minimum distance, maximum distance, and average distance:

(1) $$\begin{array}{c} d_{\min}\left(C_{i},C_{j}\right)=\underset{x\in C_{i},z\in C_{j}}{\min}\text{dist}\left(x,z\right),\\ d_{\max}\left(C_{i},C_{j}\right)=\underset{x\in C_{i},z\in C_{j}}{\max}\text{dist}\left(x,z\right),\\ d_{avg}\left(C_{i},C_{j}\right)=\frac{1}{\left|C_{i}\right|\left|C_{j}\right|}\sum_{x\in C_{i}}\sum_{z\in C_{j}}\text{dist}\left(x,z\right). \end{array}$$

The researchers optimized hierarchical clustering and proposed algorithms such as BIRCH and CURE. Each node of a cluster feature tree consists of three cluster features, including the number of samples, the vector of sample points, and the sum of squares of the sample point features [16]. The CURE algorithm reduces the effect of noise on clustering and optimizes the hierarchical clustering algorithm by choosing a fixed number of representative points to represent the class.

#### 2.1.2. Nearby Propagation Clusters

In the AP algorithm, the representative points of the class are selected from the data points.

(2) $$\begin{array}{c} z=\sum_{i=1}^{n}s\left(x_{i},x_{k}\right), \end{array}$$

where *x*_*i*_ data point is the representative point of the data *x*_*k*_ and s(*x*_*i*_, *x*_*k*_) is the similarity between the two points. In the neighbor propagation clustering algorithm, select representative points from the data points:

(3) $$\begin{array}{c} s\left(i,j\right)=-\left\|x_{i}-x_{j}\right\|, \end{array}$$

where *x*_*i*_ and *x*_*j*_ are data points.

The degree of attraction *r*(*i*, *k*) indicates the accumulation of information to consider other potential representative points *x*_*i*_*x*_*k*_, indicating the *x*_*k*_*x*_*i*_ appropriate degree of representation as a representative point.

The attractiveness *r*(*i*, *k*) indicates the appropriate degree of accumulation of information as a representative point, taking into account other potential representative points.

(4) $$\begin{array}{c} r\left(i,k\right)=s\left(i,k\right)-\underset{k^{\prime }\neq k}{\max}\left\{a\left(i,k^{\prime }\right)+s\left(i,k^{\prime }\right)\right\}. \end{array}$$

The degree of attribution *a*(*i*, *k*′) represents the appropriate degree to select a representative point as a representative point, taking into account other potential representative points. The algorithm iteratively updates the values of *r*(*i*, *k*) and *a*(*i*, *k*′) to find representative points for the data points [17]. The formula is as follows:

(5) $$\begin{array}{c} a\left(i,k\right)=\left\{\begin{array}{c} \min\left\{0,r\left(k,k\right)+\sum_{i^{\prime }\notin \left\{i,k\right\}}\max\left\{0,r\left(i^{\prime },k\right)\right\}\right\},\;i\neq k,\\ \sum_{i^{\prime }\notin \left\{i,k\right\}}\max\left\{0,r\left(i^{\prime },k\right)\right\},\;i=k. \end{array}\right. \end{array}$$

The AP algorithm describes the probability that a data point becomes a representative point by the degree of preference (preference) *p* = *s*(*k*, *k*). The larger the *p* value, the more likely the point is to become a representative point.

The attraction matrix *r* and attribution matrix *a* are initialized to a zero matrix and then selected in the order in which the attraction is updated first, and then the attribution is updated. After each round of updates, the choice of representative points is judged in a combination of attractiveness and attribution. The algorithm stops when the class boundary is updated or the generation number is reached. Another parameter in the neighbor propagation algorithm is the damping factor. In each generation, the updated results of the information are obtained by multiplying the results of the previous update by the sum of 1 of the values updated by this update. The damping coefficient avoids numerical oscillations and is used to control the convergence effect of the algorithm. The value range is [0, 1], usually set to 0.5.

(6) $$\begin{array}{c} r_{t+1}\left(i,k\right)=\lambda *r_{t}\left(i,k\right)+\left(1-\lambda \right)*r_{t+1}\left(i,k\right),\\ a_{t+1}\left(i,k\right)=\lambda *a_{t}\left(i,k\right)+\left(1-\lambda \right)*a_{t+1}\left(i,k\right). \end{array}$$

The algorithm has no requirements for the symmetry of the similarity matrix. The algorithm uses a wider range of application scenarios, clustering according to the degree of preference, and there is no need to know the number of clusters in advance. Useful when clustering cannot be scoped based on prior knowledge.

#### 2.1.3. FastText Model

The model structure is shown in Figure 1. The structure of the FastText model is similar to CBOW. The model sums word vectors in the hidden layer by mapping words in the document to the vector input hidden layer. Unlike CBOW, the output layer changes from output intermediate to output classification labels [18].

*N*-gram features describe local word order and preserve morphological features within the vocabulary. The FastText model extracts the *N*-gram characteristics of words in sentences. Since storing *N*-gram features consumes a lot of storage space, the model uses a hash function to map feature vectors, record them as input layer inputs, and then map feature vectors to the *n*-dimensional hidden layer by linear transformation. The model uses hierarchical softmax to calculate the probability distribution of a predefined class, with the goal of minimizing the value of the log-likelihood function as follows:

(7) $$\begin{array}{c} L=-N\sum_{n=1}^{N}y_{n}\log\left(f\left(BAx_{n}\right)\right), \end{array}$$

where *x*_*n*_ denote the standardized document feature vectors are *y*_*n*_ classification labels and *A* and *B* are the weight matrices.

If there are many text classification tags, the calculation cost of using softmax directly is relatively high. Therefore, the model uses hierarchical softmax to transform the global multiclassification problem into multiple binary classification problems by building a Huffman tree, thereby reducing the computational training complexity from *I*(*kh*) to *O*(*kh*). At the same time, the use of hierarchical softmax also improves the speed of the model in use.

### 2.2. Keyword Extraction Techniques

TextRank is a graph-based unsupervised text sorting model that is widely used in the field of text summary and keyword generation. The advantages of TextRank include the fact that there is no need to study documentation beforehand, and implementation is simple. The main idea is to divide the document with words or sentences and to use the divided words or sentences as nodes to construct the network diagram. Node points are connected to each other according to the similarity relationship, and the weight of the edge is the similarity between nodes. The weights of the nodes are updated iteratively, resulting in keywords or abstract sentences [19] depending on the size of node weights. The TexTank model builds a graph with a rightward figure of *G* = (*V*, *E*), where *V* is the node set, *E* is the edge set, and *E* is a subset of *x*. The weight of the sum of any two points in the figure, which indicates the degree of similarity between the two points, *W*_*ij*_  =  *W*_*ji*_.

The *V*_*i*_ score for points is calculated as

(8) $$\begin{array}{c} S\left(V_{i}\right)=\left(1-\alpha \right)+\alpha \sum_{V_{j}\in \text{ in }\left(V_{i}\right)}\frac{W_{ij}}{\sum_{V_{k}\in \text{ out }\left(V_{i}\right)}W_{jk}}s\left(V_{j}\right), \end{array}$$

where (*V*_*i*_) is the node set that points to the point and out(*V*_*i*_) is the node set that points to the node. *α* is a damping factor, with a value range of [0, 1], which indicates the probability that a node points to another node, and a typical value of 0.85.

## 3. Neural Network Model Based on Adjusting Loss Function

### 3.1. Deep Neural Network Model Construction

The overall steps of vectorized data processing and model building are shown in Figure 2.

The feed-forward neural network model framework is shown in Figure 3.

(1) Text vector calculation $\hat{y}$: because the feed-forward neural network only receives the numerical tensor, requiring the continuity of vector values, in the data processing stage before the input classifier, it is necessary to distribute words, convert them into a continuous numerical vector, then numerically calculate the word vector corresponding to each word in the sentence, convert each comment text into a large vector, and enter it into the classifier for processing for the last time. The most commonly used method of text vector calculation is the direct averaging method of word vector, that is, after text data is segmented, the word vector training is performed on each word through the word2vec model, then the corresponding word vector of each word is added, and then the corresponding position is averaged to obtain a vectorized representation of each comment data [20]. This approach means that all words in a text are considered equally important, and it may not be possible to exclude the effects of words that have little impact on the classification result. Use the text parting tool Jeba to segment preprocessed text, while removing stop words, and train by the word2vec model. Get the *N*-dimensional word vector for each word *V*_*i*_ (the total number of words is set to *W*), *V*_*i*_ = (*v*_1_, *v*_2_,…, *v*_*N*_) ∈ (1, 2,…, *M*), and for each piece of the text *D*_*j*_ (*j* = 1, 2,…, *M*), *M* represents the number of text data bars. Calculating the TF-IDF weight *T*(*t*, *D*) of each word and the number of words *n*, the final vectorization of each text is expressed as
  (9) $$\begin{array}{c} v_{j}=\frac{\sum_{t\in D_{j}}V_{t}\times T\left(t,D_{j}\right)}{n_{j}}. \end{array}$$
(2) A hidden layer neural network maps an input (text vector) to a target (label) through a series of simple data transformations (layers). The learning process is to find a set of weight values for all layers of the neural network, so that the network can vectorize the text data corresponding to each input and its correct target output value one by one [21], and the distributed text vector is input to the hidden layer, the output of the feed-forward network of the first hidden layer has the following form:
  (10) $$\begin{array}{c} NN_{MLP1}\left(v\right)=g\left(v\cdot W+b\right). \end{array}$$
(3) where *v* ∈ *R*^*d*_in_^, *W* ∈ *R*^*d*_in_*d*_out_^, and *b* ∈ *R*^*d*_out_^. *W* and *b* are the weight matrix and the bias term, respectively, and *g* is activation function.
(4) The disadvantage of the tanh function is that when the input value is very large or very small, the derivative will approach 0, making the gradient update very slow, causing the gradient to disappear. The Remu function is a piecewise linear function in the form:
  (11) $$\begin{array}{c} a\left(z\right)=\max\left(0,z\right). \end{array}$$
(5) The advantage of the Remu function is that the computation speed is fast, and it compensates for the disappearance of the gradient of the tanh function. The next calculation of the second layer also follows the transformation from above.
(6) Output layer: for the problem for multiclassification problems, the neural network is utilized. The softmax transform converts it to a probability distribution:

(12) $$\begin{array}{c} p_{i}=\text{softmax}\left(a_{i}\right)=\frac{\exp\left(a_{i}\right)}{\sum_{i=1}^{c}\exp\left(a_{i}\right)}. \end{array}$$

### 3.2. Improved Loss Function

The data transformation operations performed by each layer of input data in the neural network are stored in the weights of that layer, and deep learning is actually looking for a set of weights for all layers of the neural network, so that the network can correspond input values of each sample to its true value one by one, which is the work of loss function of the neural network. The neural network uses this distance value to adjust weights to reduce the current corresponding loss value,as shown in Figure 4.

For classification problems, the magnitude of the error between the predicted and true values is measured using loss function in the neural network, and weight parameters in the network are updated with each training of the model, with the ultimate training goal of minimizing this error [22]. For different problems, it is necessary to define loss function according to actual situation, for example, some classification problems in the real scene belong to multiple classifications, and it is necessary to construct multiclassification loss function, and for example, some data have distribution imbalance problems, and the sample weight or classification difficulty problem in loss function needs to be considered. The cross-entropy loss function of the two classes are as follows:

(13) $$\begin{array}{c} L=\left\{\begin{array}{c} -\log\;p,\text{ if }y=1,\\ -\log\left(1-p\right),\text{ otherwise.} \end{array}\right. \end{array}$$

The problem of categorical imbalance is also a manifestation of difference in classification difficulty. Thus, in the loss function of a neural network, by reducing the weights of the easier to classify samples, the model can focus more on the difficult to classify samples. Lin et al. proposed that focus loss aims to solve the problem of category imbalance in binary classification:

(14) $$\begin{array}{c} L_{\hbar }=\left\{\begin{array}{c} -{\left(1-p\right)}^{\gamma }\log\;p,\text{ if }y=1,\\ -p^{\gamma }\log\left(1-p\right),\text{ otherwise,} \end{array}\right. \end{array}$$

where *p* is the probability that the model estimates that the sample belongs to the true category. For modulation coefficients, when samples are correctly classified, modulation coefficients are relatively small and contribute less to the total loss, that is, modulation coefficient reduces loss contribution of easily divided samples, so that the model focuses on correcting misclassified samples. *γ* is a constant greater than or equal to zero that determines the magnitude of modulation coefficient's role in the loss, the greater the modulation coefficient's effect, and when *γ*  = 0, the focal loss is equivalent to the cross-entropy loss [23].

In addition, the researchers found following weight adjustments for the focus loss, and the experimental results showed a slight improvement:

(15) $$\begin{array}{c} L_{\hbar }=\left\{\begin{array}{c} -\alpha \cdot {\left(1-p\right)}^{\gamma }\log\;p,\text{ if }y=1,\\ -\left(1-\alpha \right)\cdot p^{\gamma }\log\left(1-p\right),\text{ otherwise}. \end{array}\right. \end{array}$$

Experimental data on Lin et al. showed that positive samples are a minority. The model works best when *α*  = 0.25 and *γ*  = 2, with the effect of modifying modulation coefficients to avoid the relatively small weights assigned to easily classified samples, which should be *γ* slightly reduced when slightly increased *α*. Now, considering the multiclassification case, traditional loss function is defined as follows:

(16) $$\begin{array}{c} L=-\sum_{c=1}^{M}y_{c}\log\left(p_{c}\right). \end{array}$$

Assuming *M* is the number of categories, it is the indicator variable, and the form of the category label *y* is one-hot. For sample *x*, if the real number category is class *c*, then the *c*th bit of the vector is 1, and the remaining bits are 0. The probability that the sample is predicted for each class is as follows: now, use the idea of focus loss to solve the multiclass problem, referring to multiclass cross-entropy loss function form, the multiclass focus loss is defined as follows:

(17) $$\begin{array}{c} L_{\hbar }=-\sum_{i=1}^{c}y_{i}\cdot {\left(1-p_{i}\right)}^{\gamma }\log\left(p_{i}\right). \end{array}$$

It converts the category label *y* of data to the form one-hot, *c* is the number of categories, and *p* is the probability that the sample will be predicted as a category. To further balance the interference caused by the sample scale, a weighted factor *a*1 can also be introduced, which is used to represent the probability that the sample predicts correctly in *p*, and *L* can also be expressed as

(18) $$\begin{array}{c} L_{\hbar }=-\alpha_{t}{\left(1-p_{t}\right)}^{\gamma }\log\left(p_{t}\right). \end{array}$$

For weight adjustment parameter *A*, if it is applied to cross-entropy loss function, it can be set to inverse frequency of each category, or the optimal value can be obtained by cross-validation. There are two parameters in the focal damage, *Y* and *A* are one and the other relationship and *A* is more of a correction effect, which need to be through the cross-validation of Lin et al. to vigorously adjust its optimal value, after adjusting the parameters. The value of a has only a slight improvement in the classification effect [24] and can be thought as 1, and loss function used by the model is shown in equation (17). In the case of using focus loss function, the forward computation process of the neural network is shown in Figure 5:

The fully connected layer *a*_*i*_ for the *i*th output, the softmax layer is later linked, the predicted probability values of each category are calculated, and the focus loss of the calculation process is updated backwards as follows:

(19) $$\begin{array}{c} \frac{\partial L_{\hbar }}{\partial a_{i}}=\left\{\begin{array}{c} -{\left(1-p_{t}\right)}^{\gamma }\cdot \left(1-p_{t}-\gamma p_{t}\log\;p_{t}\right),\;i=t,\\ p_{i}\cdot {\left(1-p_{t}\right)}^{\gamma -1}\cdot \left(1-p_{t}-\gamma p_{t}\log\;p_{t}\right),\;i\neq t. \end{array}\right. \end{array}$$

## 4. Experimental and Algorithmic Evaluation Depth Prices

### 4.1. Experimental Evaluation Indicators

Overall, the model is more accurate in its evaluation metrics in the field of text sentiment analysis (accuracy) and recall. They all represent different performances, but the same is that the higher the value, the better the performance of the classifier.

The above evaluation criteria are generally used for binary classification problems, and data sets used in the experimental section of this chapter clearly indicate that multiple categories will be identified; so based on this consideration, the evaluation criteria under this type will be described as follows. Considering the multicategory problem as a number of binary classification problems, assuming that a certain text data can be clearly distinguished into three categories *A*, *B*, and *C*, then for the research object, a class, there is an elephant Table 1. This is a kind of confusion matrix.

Therefore, the calculation formula for each evaluation criterion is as follows: accuracy, Acc:

(20) $$\begin{array}{c} \text{Acc}=\frac{\text{TA}+\text{TNA}}{\text{TA}+\text{FA}+\text{FNA}+\text{TNA}}. \end{array}$$

Precision, *P*:

(21) $$\begin{array}{c} P=\frac{\text{TA}}{\text{TA}+\text{FA}}. \end{array}$$

Recall, *R*:

(22) $$\begin{array}{c} R=\frac{\text{TA}}{\text{TA}+\text{FNA}}. \end{array}$$

*F*1 value:

(23) $$\begin{array}{c} F1=\frac{2\times P\times R}{P+R}. \end{array}$$

We assume that *n* categories need to be evaluated, a total of *N* samples, and exactly match the number of categories, so this article will calculate the mean of the above evaluation criteria as an evaluation criterion, as follows:

(24) $$\begin{array}{c} {\text{Acc}}_{\text{avg}}=\frac{1}{N}\sum \left(\text{Acc}*m_{i}\right). \end{array}$$

Similarly,

(25) $$\begin{array}{c} P_{\text{avg}}=\frac{1}{N}\sum \left(P_{i}*m_{i}\right),\\ R_{\text{avg}}=\frac{1}{N}\sum \left(R_{i}*m_{i}\right),\\ F1_{\text{avg}}=\frac{1}{N}\sum \left(F1_{i}*m_{i}\right). \end{array}$$

### 4.2. Model Training Process

When training the HCB model constructed in this paper, it is clear that some params settings affect the classification results, and in this section, the experiments in question eventually identify the params of some nodes. In this article, we need to use the relevant evaluation indicators to evaluate the performance of the model, and the following will build the model for some experiments and training. Among them, the training takes the form of setting parameters, as shown in Tables 1–3, to obtain parameters that contribute to the excellent performance of the model.

From Figures 6 and 7, it can be seen that the HCB model constructed in this paper is relatively stable, and final loss function tends to a value, indicating convergence, and the model can be used for classification. In addition, changes in Acc indicate that the model performs well.

In the previous settings of params, the selection of word vector models and the setting of word vector dimensions were ignored. These two cannot simply be subjective and need to be clarified by experimentation. Therefore, the following experiment is to obtain the orientation of two models for the built model HCB at different sizes. Use only Acc as an evaluation criterion to obtain the experimental results plot as shown in Figure 8.

As can be seen from this comparison result, for the HC model constructed in this paper, the word vector dimension obtained by the 200 word2vec and Glore models performed better, and the word vector obtained by the word2vec model was better than others. Thus, fix the word vector dimensions and model of the model in the following experimental section.

### 4.3. Experimental Results

The CNN and BiLSTM models involved in the literature were selected to classify the first dataset mentioned in this paper, and the final results are shown in Figure 9.

According to the experimental comparison results, the results of two typical classification models are not very poor. Obviously, the classification effect of CNN is better than that of BiLSTM, reflecting the effectiveness of the HCB model.

In this paper, the comparison experiment is based on the real value. The experimental results shown in Figure 10 show that the LSTM model is highly accurate.

By using a prediction method based on support vector machine, this paper verifies whether the topic heat trend prediction model based on LSTM has a high degree of reduction over time, and the experimental results are shown in Figure 11.

From the above figure, it can be seen that the average error on the test set is 0.08342, and the topic heat trend prediction model based on LSTM is more in line with the real situation, reflecting the rationality and superiority of the proposed model.

## 5. Conclusion

Internet information exchange has become the mainstream of modern social networking, the real-time, accuracy, traceability, and reliability of Internet communication, so that the public relies on it to disseminate and obtain information. The Internet communication platform has gradually become a distribution center of social opinion, through the deep excavation of the topic, you can find the development law of the topic, convenient for users to track interest and personalized experience. In this paper, the embedded matrix is constructed as the input of the CNN-GRU model through data preprocessing, word frequency statistical analysis, and text vectorization, and then the loss function is improved to improve the classification effect of the model on the small category data to alleviate the data imbalance; finally, combined with the deep neural network model proposed in this paper, several sets of comparative experiments are designed to prove the improvement of classification performance of the model and the effectiveness of the optimized model.

At present, it is based on the real user data of Xinlang Weibo, which has strong authority. Follow-up research work will focus on the following points:

1. Increase the extraction rate of seat features to improve the accuracy of hotspot recognition
2. The classification of hot topics is complex, and the classification of hot topics and the prediction of hot development trends by category can improve the prediction efficiency

## Figures and Tables

**Figure 1:** FastText structure diagram.

**Figure 2:** Schematic diagram of model building.

**Figure 3:** Feed-forward neural network construction.

**Figure 4:** The process by which a neural network implements predictions.

**Figure 5:** Forward computation of the neural network under focus loss.

**Figure 6:** Loss change during training.

**Figure 7:** Acc change graph during training.

**Figure 8:** Word vector dimension comparison chart.

**Figure 9:** Comparison of CNN and BiLSTM models' training results.

**Figure 10:** Comparison of the predicted value and the true value of the topic heat trend prediction model based on LSTM.

**Figure 11:** Comparison of prediction results.

**Table 1:** Convolutional module parameter setting table.

The parameter name	Convolutional kernel size	Number of convolutional kernels	*K* value of pooling
Value	3, 4, 5	128	3

**Table 2:** Cyclic module parameter setting table.

The parameter name	The number of nodes hidden by BiLSTM	Attention dimension
Value	256	512

**Table 3:** HCB model parameter settings.

The parameter name	The parameter value
Embed layer dropout values	0.2
Full-connection layer dropout value	0.2
Optimizer	AdaGrad
Number of trainings	50
Learning rate	0.01
Batch_size	64
The number of nodes in the fully connected tier	256

## Data Availability

The experimental data used to support the findings of this study are available from the corresponding author upon request.
